The article "Estimations of Generalized Exponential Distribution Parameters Based on Type I Generalized Progressive Hybrid Censored Data" was published in 2022. Journal: Comput Math Methods Med.

# Estimations of Generalized Exponential Distribution Parameters Based on Type I Generalized Progressive Hybrid Censored Data

**DOI:** 10.1155/2022/8058473

**Published:** 2022-03-29

**Authors:** M. Nagy, Adel Fahad Alrasheedi

**Affiliations:** Department of Statistics and Operations Research, College of Science, King Saud University, P.O. Box 2455, Riyadh 11451, Saudi Arabia

## Abstract

Type I generalized progressive hybrid censoring scheme is a combination of Type I and Type II progressive hybrid censoring schemes, and it is one of the most recent advancements in data censoring. In this article, based on Type I generalized progressive hybrid censoring data from generalized exponential distribution, the maximum likelihood and Bayesian estimators of distribution's parameters as well as the reliability and hazard functions are approximately calculated. Also, the credible interval estimators of these quantities are obtained. Since these quantities cannot be obtained in closed form, so simulation and analysis using a Monte Carlo simulation study with Gibbs sampling are taken. Finally, an illustrative example using real data set is presented to compare the proposed procedures presented and developed here.

## 1. Introduction

Computational methods and data processing are among the most important sciences that have different applications in many fields such as medicine, engineering, agriculture, and various vital fields. For a large data, it was necessary to find method for statistical inference by using small samples taken in a certain way of this large data, in order to limit the time and the cost; hence, the idea of censored samples started. There are a variety of scenarios where observed data is censored in nature, including reliability and life testing experiments. The two most popular censoring techniques are Type I and Type II censoring schemes. Epstein [1] initially proposed the hybrid censoring scheme, which is a mixture of Type I and Type II censoring schemes. One of the main problems of Type I, Type II, and hybrid censoring (HC) methods is that they do not allow for unit removal at whatever point other than the experiment's finish. To address this issue, a more comprehensive censoring scheme known as progressive Type II censoring was implemented. Balakrishnan and Cramer [2] provide a full discussion of these censoring schemes as well as some recent advances. The disadvantages of the progressive Type II censoring scheme are that the time of the experiment can be very long if the units are highly reliable. Therefore, Kundu and Joarder [3] proposed a progressive hybrid censoring scheme (PHCS). Under progressive hybrid censoring scheme, the time on experiment will be no more than *T*. Some recent studies on progressive hybrid censoring have been carried out by many authors including Lin et al. [4], Panahi [5], Mohie El-Din et al. [6], and El-Din et al. [7]. On the other side, one of the progressive hybrid censoring scheme's drawbacks is that it cannot be used when there are only a few failures before time *T*.

The article "Estimations of Generalized Exponential Distribution Parameters Based on Type I Generalized Progressive Hybrid Censored Data" was published in 2022. Journal: Comput Math Methods Med.

Cho et al. [8] suggest a Type I generalized PHCS that allows us to notice a prespecified number of failures for this reason. As a result, a specified number of failures and their lifetimes are always supplied under the Type I generalized PHCS. The life testing experiment based on this censoring scheme can reduce total test duration as well as the cost incurred due to unit failures. Furthermore, because there are more failed observations, statistical estimating efficiency improves. The Type I generalized PHCS have been investigated for instance by El-Din et al. [9], Nagy et al. [10, 11], and Nagy and Alrasheedi [12].

We look at statistical inference for a generalized exponential (GE) distribution under Type I generalized PHCS in this paper. Gupta and Kundu [13] provide the probability density function (PDF) and cumulative distribution function (CDF) of the GE distribution, respectively.

(1) $$\begin{array}{c} f\left(x;\alpha ,\lambda \right)=\alpha \lambda \exp\left(-\lambda x\right){\left[1-\exp\left(-\lambda x\right)\right]}^{\alpha -1},\;x,\alpha ,\lambda >0, \end{array}$$

(2) $$\begin{array}{c} F\left(x;\alpha ,\lambda \right)={\left[1-\exp\left(-\lambda x\right)\right]}^{\alpha },\;x,\alpha ,\lambda >0, \end{array}$$

where *α* and *λ* denote the shape and scale parameters, respectively. For simplicity, let *ψ*(*x*; *λ*) = 1 − exp(−*λx*); then, PDF and CDF of the GE distribution can be rewritten, respectively, by the following:

(3) $$\begin{array}{c} f\left(x;\alpha ,\lambda \right)=\alpha \lambda \exp\left(-\lambda x\right){\left[\psi \left(x;\lambda \right)\right]}^{\alpha -1},\;x,\alpha ,\lambda >0, \end{array}$$

(4) $$\begin{array}{c} F\left(x;\alpha ,\lambda \right)={\left[\psi \left(x;\lambda \right)\right]}^{\alpha },\;x,\alpha ,\lambda >0. \end{array}$$

Therefore, the reliability (survival) and hazard functions may be written, respectively, as follows:

(5) $$\begin{array}{c} S\left(x;\alpha ,\lambda \right)=1-{\left[\psi \left(x;\lambda \right)\right]}^{\alpha },\;x,\alpha ,\lambda >0, \end{array}$$

(6) $$\begin{array}{c} H\left(x;\alpha ,\lambda \right)=\frac{f\left(x;\alpha ,\lambda \right)}{S\left(x;\alpha ,\lambda \right)}=\frac{\alpha \lambda \exp\left(-\lambda x\right){\left[\psi \left(x;\lambda \right)\right]}^{\alpha -1}}{1-{\left[\psi \left(x;\lambda \right)\right]}^{\alpha }},\;x,\alpha ,\lambda >0. \end{array}$$

The GE distribution is a very flexible and favorably skewed model that is used to replace the lognormal, gamma, and Weibull distributions. It is often used to examine data that is skewed in a positive direction. Inferences for the GE distribution have been discussed by many authors including Gupta and Kundu [14] and Jaheen [15].

The article "Estimations of Generalized Exponential Distribution Parameters Based on Type I Generalized Progressive Hybrid Censored Data" was published in 2022. Journal: Comput Math Methods Med.

The aim of this article is that we consider the analysis of the Type I progressive censoring data from generalized exponential distribution to calculate the maximum likelihood and Bayesian estimators of unknown parameters and also calculate the approximate confidence intervals. The remainder of this paper is as follows. In Section 2, we provide an overview of the Type I generalized PHCS and compute the likelihood function of the model based on Type I generalized PHCS. The ML estimators with the corresponding approximate confidence intervals of the GE distribution's parameters, the reliability function and hazard function, are derived in Section 3. In Section 4, we use MCMC with the Gibbs sampling procedure to compute the Bayesian estimates of the parameters, reliability and hazard functions for the GE distribution, and also construct their credible intervals. Under Type I generalized censoring scheme, simulation studies to compare the efficacy of the offered inference methodologies are carried out in Section 5. In Section 6, some computational results with real data are presented for illustrating all the inferential methods developed here. Finally, Section 7 concludes the paper.

## 2. The Likelihood Model Description

Consider life testing experiment in which *n* equivalent units are tested. For *T* ∈ (0, ∞) and integers *k*, *m* ∈ {1, 2, ⋯, *n*} and *R* = (*R*_1_, ⋯−*R*_*m*_) are prefixed such that *k* < *m*. Let *d* denote the number of observed failures up to time *T*, and *Y*_*k*:*m*:*n*_ and *Y*_*m*:*m*:*n*_ are the times of failure *k*, *m*, respectively. According to the Type I generalized PHCS which introduced by Cho et al. [8], the experiment termination time is *T*^∗^ = max{*Y*_*k*:*m*:*n*_, min{*Y*_*m*:*m*:*n*_, *T*}}  and we have the following observations:

1. Suppose *T* is reached before the *k*^th^ failure, then the experiment terminates at *Y*_*k*:*m*:*n*_ and we will observe {*Y*_1:*m*:*n*_<⋯<*Y*_*d*:*m*:*n*_ < *Y*_*d*+1:*m*:*n*_<⋯<*Y*_*k*:*m*:*n*_}
2. Suppose that the *T* is reached between the *k*^th^ and *m*^th^, then the experiment terminates at *T* and we will observe {*Y*_1:*m*:*n*_<⋯<*Y*_*k*:*m*:*n*_ < *Y*_*k*+1:*m*:*n*_<⋯<*Y*_*D*:*m*:*n*_}
3. Suppose that the *m*^th^ failure occurs before *T* (i.e., *Y*_*m*:*m*:*n*_ ≤ *T*), then the experiment terminates at *X*_*m*:*m*:*n*_ and we will observe {*Y*_1:*m*:*n*_<⋯<*Y*_*k*:*m*:*n*_ < *Y*_*k*+1:*m*:*n*_<⋯<*Y*_*m*:*m*:*n*_}

Thus, the joint density function based on the above cases can be written as follows:

(7) $$\begin{array}{c} f\left(\underline{Y}\right)=C_{i,j}\left[\overset{D^{*}}{\underset{i=1}{\prod }}f\left(y_{i:m:n}\right){\left[S\left(y_{i:m:n}\right)\right]}^{R_{i}^{*}}\right]{\left[S\left(T\right)\right]}^{R_{\tau }^{*}}, \end{array}$$

where

(8) $$\begin{array}{c} C_{i,j}=\left[\overset{D^{*}}{\underset{i=1}{\prod }}\overset{m}{\underset{j=1}{\sum }}R_{j}^{*}\right],\\ D^{*}=\max\left\{k,\min\left\{m,d\right\}\right\},\\ R^{*}=\left\{\begin{array}{cc} \left(R_{1},\cdots ,R_{d},\cdots ,R_{k}\right), & \text{if }T<Y_{k:m:n},\\ \left(R_{1},\cdots ,R_{k},\cdots ,R_{d}\right), & \text{if }Y_{k:m:n}<T<Y_{m:m:n},\\ \left(R_{1},\cdots ,R_{k},\cdots ,R_{m}\right), & \text{if }Y_{k:m:n}<T, \end{array}\right. \end{array}$$

where *R*_*τ*_^∗^ is the number of surviving units eliminated at *T*, as determined by the following:

(9) $$\begin{array}{c} R_{\tau }^{*}=\left\{\begin{array}{cc} 0, & \text{if }T<Y_{k:m:n},\\ \overset{d}{\underset{j=1}{\sum }}R_{j}, & \text{if }Y_{k:m:n}<T<Y_{m:m:n},\\ 0, & \text{if }Y_{k:m:n}<T, \end{array}\right. \end{array}$$

with

(10) $$\begin{array}{c} \underline{y}=\left\{\begin{array}{cc} \left(y_{1},\cdots ,y_{d},\cdots ,y_{k}\right), & \text{if }T<Y_{k:m:n},\\ \left(y_{1},\cdots ,y_{k},\cdots ,y_{d}\right), & \text{if }Y_{k:m:n}<T<Y_{m:m:n},\\ \left(y_{1},\cdots ,y_{k},\cdots ,y_{m}\right), & \text{if }Y_{k:m:n}<T, \end{array}\right. \end{array}$$

and *x*_*i*_ = *x*_*i*:*m*:*n*_ for simplicity of notation.

The article "Estimations of Generalized Exponential Distribution Parameters Based on Type I Generalized Progressive Hybrid Censored Data" was published in 2022. Journal: Comput Math Methods Med.

Upon using Equations (3) and (4) in Equation (7), the likelihood function of *α*, *β* based on generalized Type I HPCS can be obtained as follows:

(11) $$\begin{array}{c} L\left(\alpha ,\lambda \;|\;\underline{y}\right)=C_{i,j}\alpha^{D^{*}}\lambda^{D^{*}}\exp\left(-\lambda \overset{D^{*}}{\underset{i=1}{\sum }}y_{i}\right)\exp\left\{\left(\alpha -1\right)\overset{D^{*}}{\underset{i=1}{\sum }}\ln\left[\psi \left(y_{i};\lambda \right)\right]\right\}\times \exp\left\{R_{\tau }^{*}\ln\left[1-{\left[\psi \left(T;\lambda \right)\right]}^{\alpha }\right]+\overset{D^{*}}{\underset{i=1}{\sum }}R_{i}^{*}\ln\left[1-{\left[\psi \left(y_{i};\lambda \right)\right]}^{\alpha }\right]\right\}. \end{array}$$

## 3. The ML Estimations

For computing the ML estimates, we must maximize the likelihood $L\left(\alpha ,\lambda |\underline{y}\right)$ with respect to *α* and *λ* in order to compute the ML estimates. The logarithm of the likelihood function is given by:

(12) $$\begin{array}{c} \ell \left(\alpha ,\lambda \;|\;\underline{y}\right)\propto D^{*}\ln\alpha +D^{*}\ln\lambda -\lambda \overset{D^{*}}{\underset{i=1}{\sum }}y_{i}+\left(\alpha -1\right)\overset{D^{*}}{\underset{i=1}{\sum }}\ln\left[\psi \left(y_{i};\lambda \right)\right]+\overset{D^{*}}{\underset{i=1}{\sum }}R_{i}^{*}\ln\left[1-{\left[\psi \left(y_{i};\lambda \right)\right]}^{\alpha }\right]+R_{\tau }^{*}\ln\left[1-{\left[\psi \left(T;\lambda \right)\right]}^{\alpha }\right]. \end{array}$$

The ML estimates ${\hat{\alpha }}_{\text{ML}}$ and ${\hat{\lambda }}_{\text{ML}}$ of *α* and *λ* can be obtained by simultaneously solving the following equations.

(13) $$\begin{array}{c} \frac{\partial \ell \left(\alpha ,\lambda \;|\;\underline{y}\right)}{\partial \alpha }=\frac{D^{*}}{\alpha }+\overset{D^{*}}{\underset{i=1}{\sum }}\ln\left[\psi \left(y_{i};\lambda \right)\right]-\overset{D^{*}}{\underset{i=1}{\sum }}R_{i}^{*}\frac{{\left[\psi \left(y_{i};\lambda \right)\right]}^{\alpha }\ln\left[\psi \left(y_{i};\lambda \right)\right]}{1-{\left[\psi \left(y_{i};\lambda \right)\right]}^{\alpha }}-R_{\tau }^{*}\frac{{\left[\psi \left(T;\lambda \right)\right]}^{\alpha }\ln\left[\psi \left(T;\lambda \right)\right]}{1-{\left[\psi \left(T;\lambda \right)\right]}^{\alpha }}=0, \end{array}$$

(14) $$\begin{array}{c} \frac{\partial \ell \left(\alpha ,\lambda \;|\;\underline{y}\right)}{\partial \lambda }=\frac{D^{*}}{\lambda }-\overset{D^{*}}{\underset{i=1}{\sum }}y_{i}+\left(\alpha -1\right)\overset{D^{*}}{\underset{i=1}{\sum }}\frac{y_{i}\left[1-\psi \left(y_{i};\lambda \right)\right]}{\psi \left(y_{i};\lambda \right)}-\alpha \overset{D^{*}}{\underset{i=1}{\sum }}R_{i}^{*}\frac{y_{i}\left[1-\psi \left(y_{i};\lambda \right)\right]{\left[\psi \left(y_{i};\lambda \right)\right]}^{\alpha }}{1-{\left[\psi \left(y_{i};\lambda \right)\right]}^{\alpha }}-\alpha R_{\tau }^{*}\frac{T\left[1-\psi \left(T;\lambda \right)\right]{\left[\psi \left(T;\lambda \right)\right]}^{\alpha }}{1-{\left[\psi \left(T;\lambda \right)\right]}^{\alpha }}=0. \end{array}$$

By using the invariance property of the ML estimator, the ML estimators of the corresponding reliability and hazard functions are given, respectively, by

(15) $$\begin{array}{c} {\hat{S}}_{\text{ML}}\left(t\right)=1-{\left[\psi \left(t;{\overset{\wedge }{\lambda }}_{\text{ML}}\right)\right]}^{{\overset{\wedge }{\alpha }}_{\text{ML}}-1},\;t>0, \end{array}$$

(16) $$\begin{array}{c} {\hat{H}}_{\text{ML}}\left(t\right)=\frac{{\hat{\alpha }}_{\text{ML}}{\hat{\lambda }}_{\text{ML}}\exp\left(-{\hat{\lambda }}_{\text{ML}}t\right){\left[\psi \left(y_{i};{\overset{\wedge }{\lambda }}_{\text{ML}}\right)\right]}^{{\overset{\wedge }{\alpha }}_{\text{ML}}-1}}{1-{\left[\psi \left(t;{\overset{\wedge }{\lambda }}_{\text{ML}}\right)\right]}^{{\overset{\wedge }{\alpha }}_{\text{ML}}}}. \end{array}$$

The article "Estimations of Generalized Exponential Distribution Parameters Based on Type I Generalized Progressive Hybrid Censored Data" was published in 2022. Journal: Comput Math Methods Med.

### 3.1. Approximate Confidence Intervals for *α* and *λ*

For large observation *D*^∗^, the observed Fisher information matrix of the parameters *α* and *λ* is given by the following:

(17) $$\begin{array}{c} I\left({\hat{\alpha }}_{\text{ML}},{\hat{\lambda }}_{\text{ML}}\right)={\left[\begin{array}{cc} -\frac{\partial^{2}\ell \left(\alpha ,\lambda \;|\;\underline{y}\right)}{\partial \alpha^{2}} & -\frac{\partial^{2}\ell \left(\alpha ,\lambda \;|\;\underline{y}\right)}{\partial \alpha \partial \lambda }\\ -\frac{\partial^{2}\ell \left(\alpha ,\lambda \;|\;\underline{y}\right)}{\partial \alpha \partial \lambda } & -\frac{\partial^{2}\ell \left(\alpha ,\lambda \;|\;\underline{y}\right)}{\partial \lambda^{2}} \end{array}\right]}_{\alpha ={\hat{\alpha }}_{\text{ML}},\lambda ={\hat{\lambda }}_{\text{ML}}}, \end{array}$$

where

(18) $$\begin{array}{c} \frac{\partial^{2}\ell \left(\alpha ,\lambda \;|\;\underline{y}\right)}{\partial \alpha^{2}}=\frac{-D^{*}}{\alpha^{2}}-\overset{D^{*}}{\underset{i=1}{\sum }}R_{i}^{*}\left\{\frac{{\left[\psi \left(y_{i};\lambda \right)\right]}^{2\alpha }\ln{\left[\psi \left(y_{i};\lambda \right)\right]}^{2}}{{\left\{1-{\left[\psi \left(y_{i};\lambda \right)\right]}^{\alpha }\right\}}^{2}}+\frac{{\left[\psi \left(y_{i};\lambda \right)\right]}^{\alpha }\ln{\left[\psi \left(y_{i};\lambda \right)\right]}^{2}}{1-{\left[\psi \left(y_{i};\lambda \right)\right]}^{\alpha }}\right\}-R_{\tau }^{*}\left\{\frac{{\left[\psi \left(T;\lambda \right)\right]}^{2\alpha }\ln{\left[\psi \left(T;\lambda \right)\right]}^{2}}{{\left\{1-{\left[\psi \left(T;\lambda \right)\right]}^{\alpha }\right\}}^{2}}+\frac{{\left[\psi \left(T;\lambda \right)\right]}^{\alpha }\ln{\left[\psi \left(T;\lambda \right)\right]}^{2}}{1-{\left[\psi \left(T;\lambda \right)\right]}^{\alpha }}\right\}, \end{array}$$

(19) $$\begin{array}{c} \frac{\partial^{2}\ell \left(\alpha ,\lambda \;|\;\underline{y}\right)}{\partial \alpha \partial \lambda }=\overset{D^{*}}{\underset{i=1}{\sum }}\frac{x_{i}\left[1-\psi \left(y_{i};\lambda \right)\right]}{\psi \left(y_{i};\lambda \right)}-\overset{D^{*}}{\underset{i=1}{\sum }}R_{i}^{*}\left\{\frac{\alpha y_{i}\left[1-\psi \left(y_{i};\lambda \right)\right]{\left[\psi \left(y_{i};\lambda \right)\right]}^{\alpha }\ln\left[\psi \left(y_{i};\lambda \right)\right]}{\psi \left(y_{i};\lambda \right)\left\{1-{\left[\psi \left(y_{i};\lambda \right)\right]}^{\alpha }\right\}}\right.+\frac{x_{i}\left[1-\psi \left(y_{i};\lambda \right)\right]{\left[\psi \left(y_{i};\lambda \right)\right]}^{\alpha }}{\psi \left(y_{i};\lambda \right)\left\{1-{\left[\psi \left(y_{i};\lambda \right)\right]}^{\alpha }\right\}}+\left.\frac{\alpha y_{i}\left[1-\psi \left(y_{i};\lambda \right)\right]{\left[\psi \left(y_{i};\lambda \right)\right]}^{2\alpha }\ln\left[\psi \left(y_{i};\lambda \right)\right]}{\psi \left(y_{i};\lambda \right){\left\{1-{\left[\psi \left(y_{i};\lambda \right)\right]}^{\alpha }\right\}}^{2}}\right\}-R_{\tau }^{*}\left\{\frac{\alpha T\left[1-\psi \left(T;\lambda \right)\right]{\left[\psi \left(T;\lambda \right)\right]}^{\alpha }\ln\left[\psi \left(T;\lambda \right)\right]}{\psi \left(T;\lambda \right)\left\{1-{\left[\psi \left(T;\lambda \right)\right]}^{\alpha }\right\}}\right.+\frac{T\left[1-\psi \left(T;\lambda \right)\right]{\left[\psi \left(T;\lambda \right)\right]}^{\alpha }}{\psi \left(T;\lambda \right)\left\{1-{\left[\psi \left(T;\lambda \right)\right]}^{\alpha }\right\}}\left.+\frac{\alpha T\left[1-\psi \left(T;\lambda \right)\right]{\left[\psi \left(T;\lambda \right)\right]}^{2\alpha }\ln\left[\psi \left(T;\lambda \right)\right]}{\psi \left(T;\lambda \right){\left\{1-{\left[\psi \left(T;\lambda \right)\right]}^{\alpha }\right\}}^{2}}\right\}, \end{array}$$

(20) $$\begin{array}{c} \frac{\partial^{2}\ell \left(\alpha ,\lambda \;|\;\underline{\text{y}}\right)}{\partial \lambda^{2}}=\frac{-m}{\lambda^{2}}-\left(\alpha -1\right)\overset{D^{*}}{\underset{i=1}{\sum }}\left\{\frac{x_{i}^{2}\left[1-\psi \left(y_{i};\lambda \right)\right]}{\psi \left(y_{i};\lambda \right)}+\frac{x_{i}^{2}{\left[1-\psi \left(y_{i};\lambda \right)\right]}^{2}}{{\left[\psi \left(y_{i};\lambda \right)\right]}^{2}}\right\}+\overset{D^{*}}{\underset{i=1}{\sum }}R_{i}^{*}\left\{\frac{\alpha y_{i}^{2}\left[1-\psi \left(y_{i};\lambda \right)\right]{\left[\psi \left(y_{i};\lambda \right)\right]}^{\alpha }}{\psi \left(y_{i};\lambda \right)\left\{1-{\left[\psi \left(T;\lambda \right)\right]}^{\alpha }\right\}}-\frac{\alpha^{2}y_{i}^{2}\left[1-\psi \left(y_{i};\lambda \right)\right]{\left[\psi \left(y_{i};\lambda \right)\right]}^{\alpha }}{{\left[\psi \left(y_{i};\lambda \right)\right]}^{2}\left\{1-{\left[\psi \left(y_{i};\lambda \right)\right]}^{\alpha }\right\}}\right.+\left.\frac{\alpha y_{i}^{2}{\left[1-\psi \left(y_{i};\lambda \right)\right]}^{2}{\left[\psi \left(y_{i};\lambda \right)\right]}^{\alpha }}{{\left[\psi \left(y_{i};\lambda \right)\right]}^{2}\left\{1-{\left[\psi \left(T;\lambda \right)\right]}^{\alpha }\right\}}-\frac{\alpha^{2}y_{i}^{2}{\left[1-\psi \left(y_{i};\lambda \right)\right]}^{2}{\left[\psi \left(y_{i};\lambda \right)\right]}^{2\alpha }}{{\left[\psi \left(y_{i};\lambda \right)\right]}^{2}{\left\{1-{\left[\psi \left(y_{i};\lambda \right)\right]}^{\alpha }\right\}}^{2}}\right\}+R_{\tau }^{*}\left\{\frac{\alpha T^{2}\left[1-\psi \left(T;\lambda \right)\right]{\left[\psi \left(x_{i};\lambda \right)\right]}^{\alpha }}{\psi \left(T;\lambda \right)\left\{1-{\left[\psi \left(T;\lambda \right)\right]}^{\alpha }\right\}}-\frac{\alpha^{2}T^{2}\left[1-\psi \left(T;\lambda \right)\right]{\left[\psi \left(T;\lambda \right)\right]}^{\alpha }}{{\left[\psi \left(T;\lambda \right)\right]}^{2}\left\{1-{\left[\psi \left(T;\lambda \right)\right]}^{\alpha }\right\}}\right.+\left.\frac{\alpha T^{2}{\left[1-\psi \left(T;\lambda \right)\right]}^{2}{\left[\psi \left(T;\lambda \right)\right]}^{\alpha }}{{\left[\psi \left(T;\lambda \right)\right]}^{2}\left\{1-{\left[\psi \left(T;\lambda \right)\right]}^{\alpha }\right\}}-\frac{\alpha^{2}T^{2}{\left[1-\psi \left(T;\lambda \right)\right]}^{2}{\left[\psi \left(T;\lambda \right)\right]}^{2\alpha }}{{\left[\psi \left(T;\lambda \right)\right]}^{2}{\left\{1-{\left[\psi \left(T;\lambda \right)\right]}^{\alpha }\right\}}^{2}}\right\}. \end{array}$$

Based on the normal approximation of the ML estimators, $\left(\hat{\alpha }-\alpha \right)/\sqrt{V\left(\hat{\alpha }\right)}$ and $\left(\hat{\lambda }-\lambda \right)/\sqrt{V\left(\hat{\lambda }\right)}$ are asymptotically normally distributed with mean 0 and variance 1; that is,

(21) $$\begin{array}{c} \frac{\hat{\alpha }-\alpha }{\sqrt{V\left(\hat{\alpha }\right)}}\sim N\left(0,1\right),\\ \frac{\hat{\lambda }-\lambda }{\sqrt{V\left(\hat{\lambda }\right)}}\sim N\left(0,1\right). \end{array}$$

Two-sided (1 − *γ*) 100% confidence intervals for *α* and *λ* are given by $\hat{\alpha }\pm Z_{\gamma /2}\sqrt{V\left(\hat{\alpha }\right)}$ and $\hat{\lambda }\pm Z_{\gamma /2}\sqrt{V\left(\hat{\lambda }\right)}$, respectively, where $V\left(\hat{\alpha }\right)$ and $V\left(\hat{\lambda }\right)$ are the asymptotic variances of $\hat{\alpha }$ and $\hat{\lambda }$, respectively, obtained by inverting the matrix $I\left({\hat{\alpha }}_{\text{ML}},{\hat{\lambda }}_{\text{ML}}\right)$, and *Z*_*γ*/2_ is the upper *γ*^th^/2 percentile of the standard normal distribution.

The article "Estimations of Generalized Exponential Distribution Parameters Based on Type I Generalized Progressive Hybrid Censored Data" was published in 2022. Journal: Comput Math Methods Med.

### 3.2. Approximate Confidence Intervals for *S*(*t*) and *H*(*t*)

In this subsection, we calculate the estimated confidence intervals for the reliability and hazard functions using the delta method proposed by Greene [16]. The delta method is a general method for calculating confidence intervals for MLE functions that are too complex to calculate the variance analytically. It creates a linear approximation of the function and then calculates the variance of the simpler linear function that can be used for large sample inference (see [17]). Let

(22) $$\begin{array}{c} M_{1}=\left(\frac{\partial S\left(t\right)}{\partial \alpha }\frac{\partial S\left(t\right)}{\partial \lambda }\right),\\ M_{2}=\left(\frac{\partial H\left(t\right)}{\partial \alpha }\frac{\partial H\left(t\right)}{\partial \lambda }\right), \end{array}$$

where

(23) $$\begin{array}{c} \frac{\partial S\left(t\right)}{\partial \alpha }=-{\left[\psi \left(t;\lambda \right)\right]}^{\alpha }\ln\left[\psi \left(t;\lambda \right)\right], \end{array}$$

(24) $$\begin{array}{c} \frac{\partial S\left(t\right)}{\partial \lambda }=\frac{t\lambda {\left[\psi \left(t;\lambda \right)\right]}^{\alpha }\left[1-\psi \left(t;\lambda \right)\right]}{\psi \left(t;\lambda \right)}, \end{array}$$

(25) $$\begin{array}{c} \frac{\partial H\left(t\right)}{\partial \alpha }=\frac{\lambda \left[1-\psi \left(t;\lambda \right)\right]{\left[\psi \left(t;\lambda \right)\right]}^{\alpha -1}+\alpha \lambda {\left[\psi \left(t;\lambda \right)\right]}^{\alpha -1}\ln\left[\psi \left(t;\lambda \right)\right]}{1-{\left[\psi \left(t;\lambda \right)\right]}^{\alpha }}+\frac{\alpha \lambda \left[1-\psi \left(t;\lambda \right)\right]{\left[\psi \left(t;\lambda \right)\right]}^{\alpha -1}\ln\left[\psi \left(t;\lambda \right)\right]}{{\left\{1-{\left[\psi \left(t;\lambda \right)\right]}^{\alpha }\right\}}^{2}}, \end{array}$$

(26) $$\begin{array}{c} \frac{\partial H\left(t\right)}{\partial \lambda }=\frac{\alpha \left[1-\psi \left(t;\lambda \right)\right]{\left[\psi \left(t;\lambda \right)\right]}^{\alpha -1}-\alpha \lambda t\left[1-\psi \left(t;\lambda \right)\right]{\left[\psi \left(t;\lambda \right)\right]}^{\alpha -1}}{1-{\left[\psi \left(t;\lambda \right)\right]}^{\alpha }}+\frac{t\lambda^{2}{\left[1-\psi \left(t;\lambda \right)\right]}^{2}{\left[\psi \left(t;\lambda \right)\right]}^{2\alpha -2}}{\psi \left(t;\lambda \right)\left\{1-{\left[\psi \left(t;\lambda \right)\right]}^{\alpha }\right\}}+\frac{\lambda \alpha^{2}t\left[1-\psi \left(t;\lambda \right)\right]{\left[\psi \left(t;\lambda \right)\right]}^{2\alpha -1}}{\psi \left(t;\lambda \right){\left\{1-{\left[\psi \left(t;\lambda \right)\right]}^{\alpha }\right\}}^{2}}. \end{array}$$

Then, the approximate estimates of $V\left(\hat{S\left(t\right)}\right)$ and $V\left(\hat{H\left(t\right)}\right)$ are given, respectively, by the following:

(27) $$\begin{array}{c} V\left(\hat{S\left(t\right)}\right)≅{\left[M_{1}^{t}I^{-1}M_{1}\right]}_{\alpha ={\hat{\alpha }}_{\text{ML}},\lambda ={\hat{\lambda }}_{\text{ML}}}, \end{array}$$

(28) $$\begin{array}{c} V\left(\hat{H\left(t\right)}\right)≅{\left[M_{2}^{t}I^{-1}M_{2}\right]}_{\alpha ={\hat{\alpha }}_{\text{ML}},\lambda ={\hat{\lambda }}_{\text{ML}}}, \end{array}$$

where *M*_1_^*t*^ and *M*_2_^*t*^ are the transposes of the matrix *M*_1_ and *M*_2_, respectively. Again, based on the normal approximation of the ML estimators, $\left(\hat{S\left(t\right)}-S\left(t\right)\right)/\sqrt{V\left(\hat{S\left(t\right)}\right)}$ and $\left(\hat{H\left(t\right)}-H\left(t\right)\right)/\sqrt{V\left(\hat{H\left(t\right)}\right)}$ are asymptotically normally distributed with mean 0 and variance 1; these results yield (1 − *γ*) 100% approximate confidence intervals for *S*(*t*) and *H*(*t*) which are given by the following.

(29) $$\begin{array}{c} \hat{S\left(t\right)}\pm Z_{\gamma /2}\sqrt{V\left(\hat{S\left(t\right)}\right)},\\ \hat{H\left(t\right)}\pm Z_{\gamma /2}\sqrt{V\left(\hat{H\left(t\right)}\right)}. \end{array}$$

For more on different types of confidence intervals, we refer our readers to Banik et al. [18] and Almonte and Kibria [19] among others.

The article "Estimations of Generalized Exponential Distribution Parameters Based on Type I Generalized Progressive Hybrid Censored Data" was published in 2022. Journal: Comput Math Methods Med.

## 4. Bayesian Estimates

In this section, we derive the Bayesian estimates of the GE distribution's parameters *α* and *λ*, based on Type I generalized HPCS data. For the Bayesian estimations, it is under the premise that both distribution's parameters *α* and *λ* are independent and have gamma prior distributions, respectively,

(30) $$\begin{array}{c} \pi \left(\alpha \right)=\frac{b_{1}^{a_{1}}}{\Gamma \left(a_{1}\right)}\alpha^{a_{1}-1}\exp\left(-\alpha b_{1}\right),\\ \pi \left(\lambda \right)=\frac{b_{2}^{a_{2}}}{\Gamma \left(a_{2}\right)}\lambda^{a_{2}-1}\exp\left(-\lambda b_{2}\right), \end{array}$$

where hyper parameters *a*_*i*_, *b*_*i*_ for all *i* = 1, 2 are the positive real constants that indicate prior knowledge of distribution's parameters; if *a*_*i*_, *b*_*i*_ for all *i* = 1, 2 are set to be equal zero, then the informative priors *π*(*α*) and *π*(*λ*) are reduced to the noninformative priors. The joint prior density of *α* and *λ* can be obtained by multiplying *π*(*α*) by *π*(*λ*) as follows:

(31) $$\begin{array}{c} \pi \left(\alpha ,\lambda \right)=\frac{b_{1}^{a_{1}}b_{2}^{a_{2}}}{\Gamma \left(a_{1}\right)\Gamma \left(a_{2}\right)}\alpha^{a_{1}-1}\lambda^{a_{2}-1}\exp\left(-\alpha b_{1}-\lambda b_{2}\right). \end{array}$$

Upon combining Equations (11) and (31), given the Type I generalized PHCS, the corresponding posterior distribution of *α*, *λ* is obtained as follows:

(32) $$\begin{array}{c} \pi^{*}\left(\alpha ,\lambda \;|\;\underline{y}\right)=\frac{L\left(\alpha ,\lambda \;|\;\underline{y}\right)\pi \left(\alpha ,\lambda \right)}{\int_{0}^{x_{0}}\int_{0}^{\infty }L\left(\alpha ,\lambda \;|\;\underline{y}\right)\pi \left(\alpha ,\lambda \right)d\alpha d\lambda }\propto \alpha^{D^{*}+a_{1}-1}\lambda^{D^{*}+a_{2}-1}\exp\left(-\lambda \overset{D^{*}}{\underset{i=1}{\sum }}y_{i}\right)\exp\left\{\left(\alpha -1\right)\overset{D^{*}}{\underset{i=1}{\sum }}\ln\left[\psi \left(y_{i};\lambda \right)\right]\right\}\times \exp\left(-\alpha b_{1}-\lambda b_{2}\right)\exp\left\{R_{\tau }^{*}\ln\left[1-{\left[\psi \left(T;\lambda \right)\right]}^{\alpha }\right]+\overset{D^{*}}{\underset{i=1}{\sum }}R_{i}^{*}\ln\left[1-{\left[\psi \left(y_{i};\lambda \right)\right]}^{\alpha }\right]\right\}. \end{array}$$

The Bayesian estimate of a parametric function *g*(*θ*) under squared error loss (SEL) function is obtained as follows:

(33) $$\begin{array}{c} {\hat{g\left(\theta \right)}}_{BS}=\int_{0}^{\infty }\int_{0}^{\infty }g\left(\theta \right)\pi^{*}\left(\alpha ,\beta \;|\;\underline{y}\right)d\alpha d\lambda . \end{array}$$

All Bayesian estimators based on the SEL function are in the form of a ratio of two integrals for which there are no closed-form solutions, so to estimate the above integrals, we must use appropriate numerical methods. To compute Bayesian estimates and build credible intervals for the distribution's parameters *α* and *λ*, we apply here the MCMC approaches. When compared to previous methods, the MCMC method gives an alternate way for parameter estimate that is more flexible. For more details about the MCMC approaches, for further details, see [20, 21].

The article "Estimations of Generalized Exponential Distribution Parameters Based on Type I Generalized Progressive Hybrid Censored Data" was published in 2022. Journal: Comput Math Methods Med.

### 4.1. The Metropolis-Hastings Algorithm within Gibbs Sampling

The Metropolis-Hastings (MH) algorithm was presented by Metropolis et al. [22] as a general Markov chain Monte Carlo (MCMC) approach, and Hastings [23] developed the MH algorithm. The MH approach can be used to generate random samples from any arbitrary complicated target distribution with any dimension that is known up to a normalizing constant. The Gibbs sampling method is a subset of the MCMC method. It can be used to produce a sequence of samples from two or more random variables' entire conditional probability distributions. Decomposing the joint posterior distribution into entire conditional distributions for each parameter and sample from them is required for Gibbs sampling. To produce a sample from the posterior density function$\;\pi^{*}\left(\alpha ,\lambda |\underline{y}\right)$, we propose utilizing the Gibbs sampling approach.

From Equation (32), the conditional posterior density function of *α* given$\;\pi^{*}\left(\alpha |\lambda ,\underline{y}\right)$ can be obtained as follows:

(34) $$\begin{array}{c} \pi^{*}\left(\alpha \;|\;\lambda ,\underline{y}\right)\propto \alpha^{D^{*}+a_{1}-1}\exp\left\{\left(\alpha -1\right)\overset{D^{*}}{\underset{i=1}{\sum }}\ln\left[\psi \left(y_{i};\lambda \right)\right]\right\}\times \exp\left\{R_{\tau }^{*}\ln\left[1-{\left[\psi \left(T;\lambda \right)\right]}^{\alpha }\right]+\overset{D^{*}}{\underset{i=1}{\sum }}R_{i}^{*}\ln\left[1-{\left[\psi \left(y_{i};\lambda \right)\right]}^{\alpha }\right]\right\}. \end{array}$$

Similarly, the conditional posterior density function of *λ* given $\pi^{*}\left(\alpha |\lambda ,\underline{y}\right)$ can be obtained as follows:

(35) $$\begin{array}{c} \pi^{*}\left(\lambda \;|\;\alpha ,\underline{y}\right)\propto \lambda^{D^{*}+a_{2}-1}\exp\left(-\lambda b_{2}\right)\exp\left(-\lambda \overset{D^{*}}{\underset{i=1}{\sum }}y_{i}\right)\exp\left\{\left(\alpha -1\right)\overset{D^{*}}{\underset{i=1}{\sum }}\ln\left[\psi \left(y_{i};\lambda \right)\right]\right\}\times \exp\left\{R_{\tau }^{*}\ln\left[1-{\left[\psi \left(T;\lambda \right)\right]}^{\alpha }\right]+\overset{D^{*}}{\underset{i=1}{\sum }}R_{i}^{*}\ln\left[1-{\left[\psi \left(y_{i};\lambda \right)\right]}^{\alpha }\right]\right\}. \end{array}$$

Furthermore, the conditional posterior distributions of *α* and *λ* in Equations (34) and (35) cannot be reduced analytically to well-known distributions; therefore, they cannot be sampled directly using usual methods, but their plots show that they are similar to normal distributions. We employ the MH technique within the Gibbs sampling scheme with normal proposal distribution to generate random numbers from these distributions. Now, we propose the following scheme for generating and deriving the posterior density functions, as well as the Bayesian estimates and credible intervals.

1. Step 1: Start with (*α*, *λ*) as $\left(\alpha_{0},\lambda_{0}\right)=\left({\hat{\alpha }}_{\text{ML}},{\hat{\lambda }}_{\text{ML}}\right)$
2. Step 2: For *i* = 1, 2, ⋯, *N*, repeat the following steps

- Set (*α*, *λ*) = (*α*_*i*−1_, *λ*_*i*−1_)
- Generate *α*_*i*_ from $\pi^{*}\left(\alpha |\lambda ,\underline{y}\right)$ given in Equation (33) with the $N\left(\alpha_{i-1},V\left(\hat{\alpha }\right)\right)$ proposal distribution
- Generate *λ*_*i*_ from $\pi^{*}\left(\lambda |\alpha ,\underline{y}\right)$ given in Equation (35) with the $N\left(\;\lambda_{i-1},V\left(\hat{\lambda }\right)\right)$ proposal distribution
- Calculate the probabilities $p_{\alpha }=\min\left\{1,\pi^{*}\left(\alpha^{\left(*\right)}|\lambda^{\left(*\right)},\underline{y}\right)/\pi^{*}\left(\alpha |\lambda ,\underline{y}\right)\right\}$
- Calculate the probabilities $p_{\lambda }=\min\left\{1,\pi^{*}\left(\lambda^{\left(*\right)}|\alpha^{\left(*\right)},\underline{y}\right)/\pi^{*}\left(\lambda |\alpha ,\underline{y}\right)\right\}$
- Set *α*_*i*_ = *α*^(∗)^ with probability *p*_*α*_; otherwise, set *α*_*i*_ = *α*
- Set *λ*_*i*_ = *λ*^(∗)^ with probability *p*_*λ*_; otherwise, set *λ*_*i*_ = *λ*
- Set *i* = *i* + 1

Finally, some initial observations of size *B*, say, are eliminated as burn-in observations from a total *N* generated observations of *α* and *λ*, and the remaining *N*‐*B* observations can be used to compute Bayesian estimates. The required Bayesian estimates of *α* under SELF are computed as follows:

(36) $$\begin{array}{c} {\hat{\alpha }}_{BS}=\frac{1}{N-B}\overset{N-B}{\underset{i=B+1}{\sum }}\alpha_{i}. \end{array}$$

The Bayesian estimate of *λ* under SELF is given by the following:

(37) $$\begin{array}{c} {\hat{\alpha }}_{BS}=\frac{1}{N-B}\overset{N-B}{\underset{i=B+1}{\sum }}\lambda_{i}. \end{array}$$

Substituting *α*_*i*_ and *λ*_*i*_ into Equations (5) and (6) to compute *S*_*i*_(*t*) and *H*_*i*_(*t*), for *i* = 1, 2, ⋯, *N*, then the Bayesian estimates of *S*(*t*) and *H*(*t*) under SELF are computed, respectively, as follows:

(38) $$\begin{array}{c} {\hat{S\left(t\right)}}_{BS}=\frac{1}{N-B}\overset{N-B}{\underset{i=B+1}{\sum }}S{\left(i\right)}_{i}, \end{array}$$

(39) $$\begin{array}{c} {\hat{H\left(t\right)}}_{BS}=\frac{1}{N-B}\overset{N-B}{\underset{i=B+1}{\sum }}H_{i}\left(i\right). \end{array}$$

This algorithm is also useful in computing credible intervals of unknown parameters. (1 − *γ*) 100% symmetric credible intervals of *α*, *λ*, *S*(*t*), and *H*(*t*) become, respectively, the following:

(40) $$\begin{array}{c} \left(\alpha_{\left[\left(N-B\right)\left(\gamma /2\right)\right]},\alpha_{\left[\left(N-B\right)\left(1-\gamma /2\right)\right]}\right), \end{array}$$

(41) $$\begin{array}{c} \left(\lambda_{\left[\left(N-B\right)\left(\gamma /2\right)\right]},\lambda_{\left[\left(N-B\right)\left(1-\gamma /2\right)\right]}\right), \end{array}$$

(42) $$\begin{array}{c} \left(S_{\left[\left(N-B\right)\left(\gamma /2\right)\right]}\left(t\right),S_{\left[\left(N-B\right)\left(1-\gamma /2\right)\right]}\right)\left(t\right), \end{array}$$

(43) $$\begin{array}{c} \left(H_{\left[\left(N-B\right)\left(\gamma /2\right)\right]}\left(t\right),H_{\left[\left(N-B\right)\left(1-\gamma /2\right)\right]}\right)\left(t\right). \end{array}$$

The article "Estimations of Generalized Exponential Distribution Parameters Based on Type I Generalized Progressive Hybrid Censored Data" was published in 2022. Journal: Comput Math Methods Med.

## 5. Simulation Study

In this section, to evaluate the performance of the proposed methods of different estimators of the parameters presented in the preceding sections, a simulation study is carried out. Without losing generality, sample of size (*n* = 60) is used for the simulation study with different sample sizes (*k*, *m*, where *m* = 2*k*) and different values of *T* and the following censoring schemes:

- Scheme 1: *R*_1_ = *R*_*k*_ = 2(*n* − *m*)/5, *R*_*m*_ = (*n* − *m*)/5.
- Scheme 2: *R*_1_ = *R*_*m*_ = 2(*n* − *m*)/5, *R*_*k*_ = (*n* − *m*)/5.
- Scheme 1: *R*_*k*_ = *R*_*m*_ = 2(*n* − *m*)/5, *R*_1_ = (*n* − *m*)/5.

We then generate Type I generalized PHCSs from a GE distribution with *α* = 2 and *λ* = 1.2. To compute the Bayesian estimates and the credible intervals using MCMC algorithm,by using the number of iterations *N* = 11,000, the ML estimates for unknown parameters *α* and *λ* have been used as initial values for running the MCMC algorithm. The first values of the generated sequences may be far from reminded converged sequences, so the first *B* = 1,000 values are removed here to avoid the effects of the initial values and the procedure repeated 1000 times. We use the informative gamma priors for the two distribution's parameters *α*, *λ* with hyper parameters *a*_1_ = *a*_2_ = 1 and *b*_1_ = *b*_2_ = 2 (prior 1) and noninformative priors with *a*_1_ = *b*_1_ = *a*_2_ = *b*_2_ = 0 (prior 2). Performance of different point estimates is compared in terms of their mean squared error (MSE) and estimate bias (EB) values for *α*, *λ*, *S*(*t*), and *H*(*t*) with *t* = 0.6, as shown in Tables 1–4, respectively. Also, the average length (AL) and coverage probability (CP) of the 95% approximate confidence intervals are displayed in Tables 5–8.

To check the convergence of MCMC samples, we provide the key diagnostic test and trace plots with posterior density plots for different parameters and censoring schemes using the three above schemes at *m* = 40 and *T* = 1.5 with prior 1 and prior 2. Figures 1, 2, 3, and 4 show the trace plot iterations for posterior densities of *α*, *λ*, *S*(*t*), and *h*(*t*), respectively. All censoring schemes are plotted in the same way, and it has been found that the trace plots of all censoring schemes converge very well.

From Tables 1–4, as expected, we observe that the Bayesian estimates computed under informative prior have smaller MSEs than the Bayesian estimates computed under noninformative prior and ML estimates. Moreover, in most cases, the MSEs are decreases with increasing sample size (*m*, *k*) with the same time *T*. Also, for the same sample sizes, the MSEs are decreases with increasing the time *T*. Furthermore, in most cases, under the scheme 1, MSEs are smaller than corresponding with scheme 2 and scheme 3.

From Tables 5–8 may be observed that the AL of Bayesian intervals with informative priors is shorter than the corresponding length of Bayesian intervals with noninformative priors; this is to be expected. As a result, if prior information is available, it should be used. Finally, there are no significance differences between the AL of ML intervals and the corresponding AL of Bayesian intervals with noninformative priors. Hence, we can say that performance of the maximum likelihood method is worse than the Bayesian method based on informative priors.

The article "Estimations of Generalized Exponential Distribution Parameters Based on Type I Generalized Progressive Hybrid Censored Data" was published in 2022. Journal: Comput Math Methods Med.

## 6. Real Data Analysis

In this section, we perform the following data analysis for illustrative purpose. The data set is from Lawless [24]. The data given here arose in tests on endurance of deep groove ball bearings. The data are the numbers of million revolutions before failure for each of the 23 ball bearings in the life test. It has been analyzed by several authors. It has been used earlier by Gupta and Kundu [14] that the two-parameter GE distribution can be used quite effectively to analyze this data set. Also, the Kolmogorov-Smirnov goodness-of-fit test with a total sample size of 23 was conducted for the GE distribution. The test statistics *D* = 0.105825 and the corresponding *p* value of 0.93511 were obtained. As a result, the data can be considered fit to the GE distribution. We have created three Type I generalized PHCS from this uncensored data set, by fixed *m* = 15, *k* = 9, and *R* = (2, 0^(7)^, 3, 0^(5)^, 3), and in different values of *T*, we have the censoring schemes as given in Table 9. The point and the 95% confidence interval estimates of the parameters *α*, *λ*, *S*(*t* = 50), and *h*(*t* = 50) using the ML and informative and noninformative priors are presented in Table 10.

## 7. Conclusions and Discussion

In this paper, using the Type I progressive hybrid censored data from generalized exponential distribution, we construct the maximum likelihood and Bayesian estimators for the distribution's parameters, and the maximum likelihood and Bayesian estimators of the reliability and hazard functions are computed. Using the delta technique, we determined the approximate confidence intervals of the reliability and hazard functions, as well as the approximate confidence intervals of the distribution's unknown parameters. Finally, we used the Markov chain Monte Carlo approach to perform a Bayesian estimate procedure and determine credible intervals. The results showed that the Bayesian estimation is more reliable than the ML estimation.

## Figures and Tables

**Figure 1:** Trace plots of 11,000 iterations of *α*.

**Figure 2:** Trace plots of 11,000 iterations of *λ*.

**Figure 3:** Trace plots of 11,000 iterations of *S*(*t* = 0.6).

**Figure 4:** Trace plots of 11,000 iterations of *S*(*t* = 0.6).

**Table 1:** The mean and MSE values of the ML and Bayesian estimates of *α*.

			ML		Bayesian			
					Prior 1		Prior 2	
(*k*, *m*, *n*)	*T*	Scheme	Mean	MSE	Mean	MSE	Mean	MSE
(15,30,60)	0.50	1	2.1255	0.4860	2.0606	0.3239	1.9908	0.3529
(20,40,60)			2.1501	0.4315	2.1299	0.2959	2.0365	0.3842
(25,50,60)			2.1636	0.2815	2.1471	0.2448	2.0499	0.2607
(15,30,60)		2	2.1863	0.3859	2.1192	0.2579	1.9817	0.2733
(20,40,60)			2.2249	0.5032	2.2217	0.2471	2.0646	0.3562
(25,50,60)			2.0489	0.2332	2.0476	0.1898	1.9453	0.1989
(15,30,60)		3	2.1356	0.3612	2.0814	0.3226	1.9816	0.3339
(20,40,60)			2.2364	0.4384	2.2313	0.3872	2.0741	0.4091
(25,50,60)			2.1430	0.2512	2.1491	0.1808	2.0083	0.1867
(15,30,60)	1.00	1	2.1600	0.4285	2.1012	0.3207	2.0706	0.3498
(20,40,60)			2.2021	0.3454	2.2408	0.2104	2.0426	0.2780
(25,50,60)			2.0801	0.2621	2.0332	0.2065	1.9571	0.2152
(15,30,60)		2	2.2459	0.6246	2.2890	0.3873	2.1173	0.4227
(20,40,60)			2.1706	0.4180	2.1867	0.2928	2.0639	0.2935
(25,50,60)			2.0408	0.2817	2.0878	0.1511	1.9569	0.2470
(15,30,60)		3	2.0641	0.4176	2.0529	0.3936	1.9282	0.4022
(20,40,60)			2.1515	0.3330	2.1366	0.2458	2.0215	0.3108
(25,50,60)			2.2139	0.3206	2.1795	0.1851	2.0784	0.2290
(15,30,60)	1.50	1	2.0989	0.2912	2.0275	0.2347	1.9301	0.2628
(20,40,60)			2.1448	0.1987	2.0942	0.1503	1.9712	0.1544
(25,50,60)			1.9933	0.1974	2.0514	0.1042	1.9506	0.1724
(15,30,60)		2	2.1719	0.6535	2.1996	0.3790	1.9704	0.3899
(20,40,60)			2.1907	0.4195	2.2318	0.2446	2.0746	0.3094
(25,50,60)			2.1820	0.3845	2.1559	0.2338	1.9989	0.2789
(15,30,60)		3	2.1772	0.4201	2.1399	0.2094	1.9230	0.2840
(20,40,60)			2.1174	0.3313	2.1083	0.1820	1.9868	0.1869
(25,50,60)			2.1132	0.2397	2.0725	0.1990	2.0277	0.2099

The article "Estimations of Generalized Exponential Distribution Parameters Based on Type I Generalized Progressive Hybrid Censored Data" was published in 2022. Journal: Comput Math Methods Med.

**Table 2:** The mean and MSE values of the ML and Bayesian estimates of *λ*.

			ML		Bayesian			
					Prior 1		Prior 2	
(*k*, *m*, *n*)	*T*	Scheme	Mean	MSE	Mean	MSE	Mean	MSE
(15,30,60)	0.50	1	1.2644	0.2104	1.3913	0.1202	1.3719	0.1846
(20,40,60)			1.1882	0.0842	1.2538	0.0566	1.2853	0.0719
(25,50,60)			1.1952	0.0519	1.2335	0.0328	1.2726	0.0358
(15,30,60)		2	1.1988	0.1582	1.3227	0.0698	1.3446	0.1050
(20,40,60)			1.1658	0.1067	1.2446	0.0554	1.2616	0.0720
(25,50,60)			1.2218	0.0713	1.2664	0.0436	1.2938	0.0632
(15,30,60)		3	1.2277	0.1558	1.3346	0.0999	1.3628	0.1513
(20,40,60)			1.1841	0.0929	1.2305	0.058	1.2965	0.0872
(25,50,60)			1.1978	0.0622	1.2302	0.0387	1.2808	0.0475
(15,30,60)	1.00	1	1.2210	0.1241	1.3210	0.0736	1.3024	0.1005
(20,40,60)			1.1483	0.0504	1.1789	0.0337	1.2270	0.037
(25,50,60)			1.2268	0.0664	1.2777	0.0407	1.3014	0.0513
(15,30,60)		2	1.1348	0.0784	1.1834	0.0522	1.2369	0.0704
(20,40,60)			1.1922	0.0689	1.2373	0.0429	1.2710	0.0662
(25,50,60)			1.2143	0.0769	1.2333	0.0398	1.2895	0.0488
(15,30,60)		3	1.2393	0.1323	1.3069	0.0919	1.3405	0.1189
(20,40,60)			1.1692	0.0546	1.2182	0.0436	1.2580	0.0541
(25,50,60)			1.1611	0.0465	1.2143	0.031	1.2258	0.0362
(15,30,60)	1.50	1	1.2094	0.1347	1.3098	0.0867	1.3212	0.1028
(20,40,60)			1.1498	0.0505	1.2108	0.0371	1.2447	0.0433
(25,50,60)			1.2418	0.0463	1.2672	0.0269	1.2970	0.0411
(15,30,60)		2	1.2122	0.1228	1.2862	0.0721	1.3610	0.1108
(20,40,60)			1.1559	0.0547	1.1895	0.0366	1.2402	0.0513
(25,50,60)			1.1583	0.069	1.2170	0.0414	1.2324	0.0454
(15,30,60)		3	1.1581	0.0929	1.2566	0.0512	1.3192	0.0865
(20,40,60)			1.1933	0.0796	1.2580	0.0418	1.2908	0.0638
(25,50,60)			1.1920	0.0486	1.2377	0.0411	1.2455	0.0470

The article "Estimations of Generalized Exponential Distribution Parameters Based on Type I Generalized Progressive Hybrid Censored Data" was published in 2022. Journal: Comput Math Methods Med.

**Table 3:** The mean and MSE values of the ML and Bayesian estimates of *S*(*t* = 0.6).

			ML		Bayesian			
					Prior 1		Prior 2	
(*k*, *m*, *n*)	*T*	Scheme	Mean	MSE	Mean	MSE	Mean	MSE
(15,30,60)	0.50	1	0.8502	0.0402	0.8558	0.0390	0.8501	0.0394
(20,40,60)			0.8460	0.0404	0.8520	0.0374	0.8422	0.0402
(25,50,60)			0.8539	0.0374	0.8573	0.0342	0.8500	0.0367
(15,30,60)		2	0.8524	0.0377	0.8581	0.0355	0.8498	0.0361
(20,40,60)			0.8495	0.0395	0.8555	0.0339	0.8480	0.0388
(25,50,60)			0.8424	0.0378	0.8474	0.0357	0.8403	0.0371
(15,30,60)		3	0.8469	0.0343	0.8554	0.0327	0.8474	0.0340
(20,40,60)			0.8545	0.0353	0.8591	0.0347	0.8516	0.0351
(25,50,60)			0.8526	0.0381	0.8568	0.0332	0.8475	0.0349
(15,30,60)	1.00	1	0.8514	0.0361	0.8560	0.0309	0.8520	0.0328
(20,40,60)			0.8487	0.0376	0.8561	0.036	0.8430	0.0368
(25,50,60)			0.8486	0.0408	0.8491	0.0384	0.8426	0.0391
(15,30,60)		2	0.8439	0.0507	0.8544	0.0473	0.8447	0.0499
(20,40,60)			0.8515	0.0367	0.8564	0.0356	0.8495	0.0359
(25,50,60)			0.8415	0.0468	0.8459	0.0399	0.8375	0.0425
(15,30,60)		3	0.8354	0.0484	0.8437	0.0465	0.8347	0.0467
(20,40,60)			0.8454	0.0409	0.8501	0.0358	0.8405	0.0388
(25,50,60)			0.8543	0.0394	0.8555	0.0376	0.8486	0.0382
(15,30,60)	1.50	1	0.8392	0.0448	0.8451	0.0415	0.8370	0.0426
(20,40,60)			0.8438	0.0376	0.8458	0.0348	0.8371	0.0364
(25,50,60)			0.8437	0.0389	0.8522	0.0355	0.8436	0.0385
(15,30,60)		2	0.8495	0.0427	0.8584	0.0386	0.8459	0.0426
(20,40,60)			0.8486	0.0395	0.8545	0.0388	0.8460	0.039
(25,50,60)			0.8464	0.0403	0.8485	0.0371	0.8365	0.0385
(15,30,60)		3	0.8444	0.0389	0.8509	0.0378	0.8392	0.0381
(20,40,60)			0.8472	0.0407	0.8522	0.0364	0.8444	0.0367
(25,50,60)			0.8467	0.0362	0.8484	0.0324	0.8436	0.0354

**Table 4:** The mean and MSE values of the ML and Bayesian estimates of *H*(*t* = 0.6).

			ML		Bayesian			
					Prior 1		Prior 2	
(*k*, *m*, *n*)	*T*	Scheme	Mean	MSE	Mean	MSE	Mean	MSE
(15,30,60)	0.50	1	0.4572	0.1080	0.4260	0.0997	0.4371	0.1041
(20,40,60)			0.4748	0.0817	0.4482	0.0806	0.4623	0.0816
(25,50,60)			0.4541	0.0759	0.4383	0.0700	0.4461	0.0712
(15,30,60)		2	0.4637	0.0962	0.4319	0.0876	0.4392	0.0896
(20,40,60)			0.4734	0.0937	0.4486	0.0851	0.4586	0.0928
(25,50,60)			0.4718	0.0746	0.4548	0.0704	0.4615	0.0714
(15,30,60)		3	0.4689	0.0836	0.4346	0.079	0.4426	0.08
(20,40,60)			0.4595	0.0797	0.4431	0.0764	0.4433	0.0776
(25,50,60)			0.4581	0.0815	0.4422	0.0731	0.4523	0.0786
(15,30,60)	1.00	1	0.4627	0.0912	0.4347	0.0819	0.4460	0.0854
(20,40,60)			0.4758	0.0762	0.4552	0.0736	0.4690	0.0737
(25,50,60)			0.4577	0.0792	0.4459	0.0765	0.4545	0.0767
(15,30,60)		2	0.4888	0.1140	0.4574	0.1006	0.4669	0.1130
(20,40,60)			0.4607	0.0716	0.4428	0.0693	0.4496	0.0696
(25,50,60)			0.4763	0.0915	0.4609	0.0829	0.4686	0.0867
(15,30,60)		3	0.4860	0.1051	0.4564	0.099	0.4676	0.1005
(20,40,60)			0.4802	0.0858	0.4583	0.0814	0.4681	0.0856
(25,50,60)			0.4618	0.0876	0.4478	0.0831	0.4587	0.0858
(15,30,60)	1.50	1	0.4911	0.1216	0.4592	0.1104	0.4689	0.1122
(20,40,60)			0.4888	0.0967	0.4723	0.0835	0.4791	0.0943
(25,50,60)			0.4651	0.0812	0.4425	0.0765	0.4531	0.0776
(15,30,60)		2	0.4640	0.0990	0.4306	0.0892	0.4396	0.0921
(20,40,60)			0.4737	0.0854	0.4554	0.0745	0.4611	0.0811
(25,50,60)			0.4801	0.0881	0.4635	0.084	0.4816	0.088
(15,30,60)		3	0.4879	0.1015	0.4555	0.0896	0.4642	0.0938
(20,40,60)			0.4713	0.0926	0.4466	0.0811	0.4581	0.0877
(25,50,60)			0.4720	0.0807	0.4576	0.0787	0.4651	0.0796

The article "Estimations of Generalized Exponential Distribution Parameters Based on Type I Generalized Progressive Hybrid Censored Data" was published in 2022. Journal: Comput Math Methods Med.

**Table 5:** The values of AL and corresponding CP of 95% confidence interval for the ML and Bayesian estimates of *α*.

			ML		Bayesian			
					Prior 1		Prior 2	
(*k*, *m*, *n*)	*T*	Scheme	AL	CP	AL	CP	AL	CP
(15,30,60)	0.50	1	2.1503	0.76	1.2485	0.94	1.2997	0.80
(20,40,60)			1.9408	0.68	1.1051	0.98	1.2134	0.70
(25,50,60)			1.7922	0.72	1.0989	0.98	1.1467	0.72
(15,30,60)		2	2.2102	0.72	1.2233	0.96	1.3401	0.74
(20,40,60)			2.0227	0.58	1.1614	0.98	1.1647	0.76
(25,50,60)			1.6797	0.70	1.0447	0.94	1.1023	0.74
(15,30,60)		3	2.1558	0.72	1.2466	0.94	1.3393	0.78
(20,40,60)			2.0401	0.52	1.1221	0.98	1.2342	0.76
(25,50,60)			1.7730	0.78	1.0967	0.98	1.1048	0.78
(15,30,60)	1.00	1	2.0843	0.76	1.2637	0.92	1.2885	0.82
(20,40,60)			1.9442	0.70	1.1219	0.98	1.1801	0.76
(25,50,60)			1.6910	0.62	1.0046	0.94	1.1009	0.84
(15,30,60)		2	2.2203	0.72	1.2274	0.94	1.3734	0.78
(20,40,60)			1.9287	0.64	1.1161	0.96	1.1525	0.78
(25,50,60)			1.6562	0.70	1.0283	0.96	1.0504	0.74
(15,30,60)		3	2.0034	0.68	1.1686	0.84	1.2709	0.68
(20,40,60)			1.8992	0.74	1.1026	0.98	1.1746	0.76
(25,50,60)			1.8219	0.76	1.0909	0.98	1.1381	0.78
(15,30,60)	1.50	1	2.0136	0.74	1.2214	0.94	1.2681	0.84
(20,40,60)			1.8781	0.80	1.1119	0.98	1.1437	0.84
(25,50,60)			1.5959	0.76	1.0456	0.98	1.1086	0.80
(15,30,60)		2	2.1374	0.72	1.2379	0.94	1.4195	0.78
(20,40,60)			1.9462	0.60	1.1432	0.96	1.2650	0.84
(25,50,60)			1.7937	0.60	1.0337	0.94	1.0520	0.80
(15,30,60)		3	2.1235	0.80	1.2394	0.98	1.3376	0.82
(20,40,60)			1.8577	0.74	1.1798	0.96	1.2803	0.82
(25,50,60)			1.7161	0.78	1.0369	0.92	1.0517	0.80

**Table 6:** The values of AL and corresponding CP of 95% confidence interval for the ML and Bayesian estimates of *λ*.

			ML		Bayesian			
					Prior 1		Prior 2	
(*k*, *m*, *n*)	*T*	Scheme	AL	CP	AL	CP	AL	CP
(15,30,60)	0.50	1	1.1877	0.80	0.9999	0.94	1.0630	0.80
(20,40,60)			0.8905	0.78	0.7766	0.92	0.8624	0.80
(25,50,60)			0.7586	0.86	0.6683	0.94	0.7108	0.90
(15,30,60)		2	1.0973	0.80	0.9808	0.90	1.0367	0.82
(20,40,60)			0.8656	0.78	0.7879	0.90	0.7986	0.82
(25,50,60)			0.7867	0.84	0.7146	0.98	0.7386	0.86
(15,30,60)		3	1.1479	0.80	0.9962	0.92	1.0916	0.84
(20,40,60)			0.8799	0.68	0.7172	0.90	0.8368	0.82
(25,50,60)			0.7619	0.86	0.6503	0.96	0.7224	0.90
(15,30,60)	1.00	1	1.0249	0.78	0.9354	0.88	0.9515	0.82
(20,40,60)			0.8063	0.82	0.6968	0.94	0.7178	0.90
(25,50,60)			0.7685	0.86	0.6999	0.96	0.7023	0.88
(15,30,60)		2	0.9557	0.82	0.8299	0.84	0.8840	0.82
(20,40,60)			0.8473	0.80	0.7411	0.92	0.7796	0.86
(25,50,60)			0.7643	0.80	0.6494	0.94	0.7267	0.84
(15,30,60)		3	1.1049	0.78	0.9263	0.94	0.9610	0.80
(20,40,60)			0.8415	0.76	0.7543	0.92	0.7598	0.88
(25,50,60)			0.7207	0.84	0.6597	0.94	0.6705	0.92
(15,30,60)	1.50	1	1.0246	0.76	0.9332	0.92	0.9386	0.86
(20,40,60)			0.8087	0.86	0.7325	0.90	0.7539	0.90
(25,50,60)			0.7768	0.88	0.6986	1.00	0.7223	0.92
(15,30,60)		2	1.0356	0.76	0.9870	0.92	1.0260	0.86
(20,40,60)			0.8169	0.84	0.7054	0.96	0.7321	0.88
(25,50,60)			0.7170	0.76	0.6541	0.90	0.6648	0.88
(15,30,60)		3	0.9983	0.82	0.9786	0.90	0.9829	0.88
(20,40,60)			0.8602	0.86	0.8237	0.94	0.8277	0.90
(25,50,60)			0.7469	0.82	0.6584	0.92	0.6835	0.84

The article "Estimations of Generalized Exponential Distribution Parameters Based on Type I Generalized Progressive Hybrid Censored Data" was published in 2022. Journal: Comput Math Methods Med.

**Table 7:** The values of AL and corresponding CP of 95% confidence interval for the ML and Bayesian estimates of *S*(*t*).

			ML		Bayesian			
					Prior 1		Prior 2	
(*k*, *m*, *n*)	*T*	Scheme	AL	CP	AL	CP	AL	CP
(15,30,60)	0.50	1	0.1545	0.96	0.1461	0.96	0.1505	0.96
(20,40,60)			0.1502	0.90	0.1474	0.98	0.1486	0.92
(25,50,60)			0.1468	0.88	0.1441	0.96	0.1442	0.92
(15,30,60)		2	0.1498	0.92	0.1454	0.98	0.1487	0.96
(20,40,60)			0.1488	0.90	0.1434	0.98	0.1457	0.94
(25,50,60)			0.1503	0.94	0.1483	0.98	0.1484	0.98
(15,30,60)		3	0.1495	0.94	0.1465	0.96	0.1476	0.94
(20,40,60)			0.1479	0.90	0.1444	0.94	0.1452	0.94
(25,50,60)			0.1479	0.94	0.1445	0.96	0.1448	0.96
(15,30,60)	1.00	1	0.1744	0.98	0.1584	1.00	0.1594	0.98
(20,40,60)			0.1564	0.94	0.1522	0.98	0.1538	0.96
(25,50,60)			0.1522	0.92	0.1494	0.92	0.1499	0.92
(15,30,60)		2	0.1598	0.90	0.1588	0.90	0.1590	0.90
(20,40,60)			0.1543	0.94	0.1521	0.98	0.1526	0.94
(25,50,60)			0.1539	0.88	0.1504	0.98	0.1521	0.94
(15,30,60)		3	0.1586	0.92	0.1563	0.94	0.1572	0.92
(20,40,60)			0.1539	0.90	0.1509	0.94	0.1514	0.92
(25,50,60)			0.1481	0.90	0.1453	0.92	0.1459	0.92
(15,30,60)	1.50	1	0.1646	0.88	0.1614	0.92	0.1627	0.90
(20,40,60)			0.1589	0.94	0.1561	0.98	0.1564	0.96
(25,50,60)			0.1520	0.90	0.1491	0.94	0.1517	0.94
(15,30,60)		2	0.1602	0.88	0.1520	0.90	0.1577	0.90
(20,40,60)			0.1556	0.94	0.1528	0.96	0.1536	0.94
(25,50,60)			0.1543	0.90	0.1504	0.96	0.1504	0.94
(15,30,60)		3	0.1581	0.94	0.1547	0.96	0.1548	0.96
(20,40,60)			0.1529	0.94	0.1507	0.98	0.1508	0.94
(25,50,60)			0.1504	0.96	0.1487	0.96	0.1490	0.96

The article "Estimations of Generalized Exponential Distribution Parameters Based on Type I Generalized Progressive Hybrid Censored Data" was published in 2022. Journal: Comput Math Methods Med.

**Table 8:** The values of AL and corresponding CP of 95% confidence interval for the ML and Bayesian estimates of *H*(*t*).

			ML		Bayesian			
					Prior 1		Prior 2	
(*k*, *m*, *n*)	*T*	Scheme	AL	CP	AL	CP	AL	CP
(15,30,60)	0.50	1	0.3453	0.82	0.1572	0.94	0.1874	0.84
(20,40,60)			0.3277	0.92	0.3224	0.96	0.3230	0.92
(25,50,60)			0.3063	0.94	0.2999	0.96	0.3005	0.94
(15,30,60)		2	0.3553	0.86	0.3505	0.94	0.3516	0.88
(20,40,60)			0.3294	0.86	0.3245	0.94	0.3251	0.92
(25,50,60)			0.3095	0.96	0.3037	0.98	0.3050	0.98
(15,30,60)		3	0.3550	0.88	0.3532	0.94	0.3540	0.94
(20,40,60)			0.3220	0.92	0.3146	0.98	0.3175	0.98
(25,50,60)			0.3077	0.94	0.3019	0.96	0.3025	0.94
(15,30,60)	1.00	1	0.3623	0.96	0.1638	0.98	0.1866	0.96
(20,40,60)			0.3387	0.96	0.1830	0.96	0.2018	0.96
(25,50,60)			0.3087	0.92	0.1805	0.98	0.1903	0.96
(15,30,60)		2	0.3868	0.90	0.3844	0.92	0.3864	0.92
(20,40,60)			0.3352	0.94	0.3291	0.98	0.3298	0.98
(25,50,60)			0.3195	0.88	0.3144	0.94	0.3162	0.92
(15,30,60)		3	0.3856	0.90	0.3720	0.92	0.3744	0.92
(20,40,60)			0.3389	0.98	0.3325	1.00	0.3333	1.00
(25,50,60)			0.3178	0.92	0.3118	0.96	0.3124	0.96
(15,30,60)	1.50	1	0.3788	0.86	0.1878	0.94	0.2167	0.90
(20,40,60)			0.3433	0.92	0.2023	0.94	0.2162	0.94
(25,50,60)			0.3087	0.92	0.1776	0.94	0.1972	0.94
(15,30,60)		2	0.3660	0.88	0.3587	0.94	0.3638	0.94
(20,40,60)			0.3430	0.96	0.3364	0.98	0.3382	0.96
(25,50,60)			0.3269	0.94	0.3207	0.96	0.3209	0.94
(15,30,60)		3	0.3790	0.98	0.3710	1.00	0.3765	0.98
(20,40,60)			0.3337	0.94	0.3280	1.00	0.3283	0.94
(25,50,60)			0.3174	0.96	0.3116	0.98	0.3121	0.96

**Table 9:** The different Type I generalized HPCS from the real data.

Scheme 1	*T* = 50
	*D* ^∗^ = 9
	*T* ^∗^ = *x*_*k*_ = 54.12
	$\underline{x}=\left(17.88,28.92,33.00,42.12,45.60,48.80,51.84,51.96,54.12\right)$
	*R* ^∗^ = (2, 0, 0, 0, 0, 0, 0, 0, 12), *R*_*τ*_^∗^ = 0
Scheme 2	*T* = 80
	*D* ^∗^ = 12
	*T* ^∗^ = *T*
	$\underline{x}=\left(17.88,28.92,33.00,42.12,45.60,48.80,51.84,51.96,54.12,55.56,67.80,68.88\right)$
	*R* ^∗^ = (2, 0, 0, 0, 0, 0, 0, 0, 3, 0, 0, 0), *R*_*τ*_^∗^ = 6
Scheme 3	*T* = 110
	*D* ^∗^ = 15
	*T* ^∗^ = *x*_*m*_ = 105.84
	$\underline{x}=\left(17.88,28.92,33.00,42.12,45.60,48.80,51.84,51.96,54.12,55.56,67.80,68.88,98.64,105.12,105.84\right)$
	*R* ^∗^ = (2, 0, 0, 0, 0, 0, 0, 0, 3, 0, 0, 0, 0, 0, 3), *R*_*τ*_^∗^ = 0

**Table 10:** The point and 95% confidence interval estimates for the ML and Bayesian estimates of *α*, *λ*, *S*(*t* = 50) , and *H*(*t* = 50).

Parameter	Scheme	ML	Bayesian		Asymp. CI	Bayesian	
			Prior 1	Prior 2		Prior 1	Prior 2
*α*	Sch. 1	4.6436	3.9703	4.3239	(2.3051,8.0601)	(2.6509,6.4481)	(2.4204,7.6571)
	Sch. 2	4.4185	3.9936	4.0892	(2.1934,8.4708)	(2.5224,6.7767)	(2.3030,8.0473)
	Sch. 3	4.4080	3.8862	3.9674	(2.1882,8.4909)	(2.5164,6.7927)	(2.2976,8.0664)
*λ*	Sch. 1	0.0295	0.0282	0.0288	(0.0143,0.0459)	(0.0152,0.0436)	(0.0146,0.0450)
	Sch. 2	0.0290	0.0278	0.0284	(0.0139,0.0434)	(0.0147,0.0412)	(0.0142,0.0425)
	Sch. 3	0.0283	0.0271	0.0277	(0.0121,0.0423)	(0.0128,0.0402)	(0.0123,0.0415)
*S*(*t* = 50)	Sch. 1	0.7015	0.6706	0.6886	(0.5772,1.0732)	(0.6350,1.0195)	(0.6119,1.0088)
	Sch. 2	0.6924	0.6817	0.6773	(0.5800,1.0722)	(0.6380,1.0186)	(0.6148,1.0079)
	Sch. 3	0.7065	0.6870	0.6813	(0.5758,1.0736)	(0.6333,1.0200)	(0.6103,1.0092)
*H*(*t* = 50)	Sch. 1	0.0173	0.0178	0.0175	(0.0095,0.0224)	(0.0105,0.0206)	(0.0106,0.0215)
	Sch. 2	0.0174	0.0172	0.0176	(0.0095,0.0224)	(0.0107,0.0208)	(0.0108,0.0213)
	Sch. 3	0.0166	0.0167	0.0172	(0.0096,0.0222)	(0.0103,0.0200)	(0.0100,0.0211)

The article "Estimations of Generalized Exponential Distribution Parameters Based on Type I Generalized Progressive Hybrid Censored Data" was published in 2022. Journal: Comput Math Methods Med.

## Data Availability

The data used to support the findings of this study are included within the article.

## References

[1] Epstein B. (1954). Truncated life tests in the exponential case. *The Annals of Mathematical Statistics*.

[2] Balakrishnan N., Cramer E. (2014). Progressive censoring: data and models. *The Art of Progressive Censoring*.

[3] Kundu D., Joarder A. (2006). Analysis of type-II progressively hybrid censored data. *Computational Statistics & Data Analysis*.

[4] Lin C. T., Ng H. K. T., Chan P. S. (2009). Statistical inference of type-II progressively hybrid censored data with Weibull lifetimes. *Communications in Statistics—Theory and Methods*.

[5] Panahi H. (2017). Estimation methods for the generalized inverted exponential distribution under type II progressively hybrid censoring with application to spreading of micro-drops data. *Communications in Mathematics and Statistics*.

[6] Mohie El-Din M. M. M., Amein M. M., Shafay A. R., Mohamed S. (2017). Estimation of generalized exponential distribution based on an adaptive progressively type-II censored sample. *Journal of Statistical Computation and Simulation*.

[7] El-Din M. M., Shafay A. R., Nagy M. (2018). Statistical inference under adaptive progressive censoring scheme. *Computational Statistics*.

[8] Cho Y., Sun H., Lee K. (2015). Exact likelihood inference for an exponential parameter under generalized progressive hybrid censoring scheme. *Statistical Methodology*.

[9] El-Din M. M., Nagy M., Abu-Moussa M. H. (2019). Estimation and prediction for Gompertz distribution under the generalized progressive hybrid censored data. *Annals of Data Science*.

[10] Nagy M., Sultan K. S., Abu-Moussa M. H. (2021). Analysis of the generalized progressive hybrid censoring from Burr type-XII lifetime model. *AIMS Mathematics*.

The article "Estimations of Generalized Exponential Distribution Parameters Based on Type I Generalized Progressive Hybrid Censored Data" was published in 2022. Journal: Comput Math Methods Med.

[11] Nagy M., Bakr M. E., Alrasheedi A. F. (2022). Analysis with applications of the generalized type-II progressive hybrid censoring sample from Burr type-XII model. *Mathematical Problems in Engineering*.

[12] Nagy M., Alrasheedi A. F. (2022). The lifetime analysis of the Weibull model based on generalized type-I progressive hybrid censoring schemes. *Mathematical Biosciences and Engineering*.

[13] Gupta R. D., Kundu D. (1999). Generalized exponential distributions. *Australian & New Zealand Journal of Statistics*.

[14] Gupta R. D., Kundu D. (2007). Generalized exponential distribution: existing results and some recent developments. *Journal of Statistical Planning and Inference*.

[15] Jaheen Z. F. (2004). Empirical Bayes inference for generalized exponential distribution based on records. *Communications in Statistics-Theory and Methods*.

[16] Greene W. H. (2003). *Econometric Analysis*.

[17] Agresti A. (2003). *Categorical Data Analysis*.

[18] Banik S., Albatineh A. N., Abu-Shawiesh M. O. A., Kibria B. M. G. (2014). Estimating the population standard deviation with confidence interval: a simulation study under skewed and symmetric conditions. *International Journal of Statistics in Medical Research*.

[19] Almonte C., Kibria B. M. G. (2009). On some classical, bootstrap and transformation confidence intervals for estimating the mean of an asymmetrical population. *Model Assisted Statistics and Applications*.

[20] Robert C. P., Casella G., Casella G. (2004). *Monte Carlo Statistical Methods*.

[21] Ahmed E. A. (2017). Estimation and prediction for the generalized inverted exponential distribution based on progressively first-failure-censored data with application. *Journal of Applied Statistics*.

[22] Metropolis N., Rosenbluth A. W., Rosenbluth M. N., Teller A. H., Teller E. (1953). Equation of state calculations by fast computing machines. *The Journal of Chemical Physics*.

[23] Hastings W. K. (1970). Monte Carlo sampling methods using Markov chains and their applications. *Biometrika*.

[24] Lawless J. F. (1982). *Statistical Models and Methods for Lifetime Data*.

